# Cardiac Magnetic Resonance Assessment of the Protective Effect of Remote Ischemic Postconditioning on Coronary Microcirculation after Reperfusion Therapy for Acute ST-Segment Elevation Myocardial Infarction

**DOI:** 10.1155/2022/5629763

**Published:** 2022-07-05

**Authors:** Chun Wu, Zhiyong Duan, Jin Shu, Yajuan Li

**Affiliations:** ^1^Department of Gerontology, Shibei Hospital of Jing'an District, Shanghai 200443, China; ^2^Department of Gerontology, Zhongshan Hospital Wusong Branch, Fudan University/Shanghai Baoshan District Wusong Central Hospital, Shanghai 200940, China

## Abstract

This study intends to evaluate the characteristics of coronary microcirculatory function in patients with myocardial infarction undergoing reperfusion and its predictive value in assessing cardiac function, myocardial activity, recovery of ventricular wall motion after infarction, and distant myocardial remodeling by cardiac magnetic resonance technique (CMRI). *Materials and Methods*. The 293 cases of patients with myocardial infarction treated in our hospital from August 2017 to August 2021 were selected as the subjects of this retrospective study, 13 cases were shed due to transfer and moving, and the rest were divided into 140 cases each in the emergency and elective groups according to emergency percutaneous coronary intervention (PCI) and elective PCI. The patients' myocardial infarct volume ventricular volume, microcirculatory obstruction volume ventricular volume, microcirculatory obstruction volume/myocardial infarct volume, and LVEF, combined with BP and troponin T, were analysed by CMR for comparative analysis, hemodynamic, and cardiac function index differences. *Results*. The hemodynamics (CO, CI, SV, SI, LVSW1, and LCW) measured at different times were significantly different between the two groups; patients in the emergency group had significantly lower EDV and ESV than the elective group at 7-10 d postoperatively; and EDV, ESV, and LVEF improved in both groups after 3 months, while EDV, ESV, and LVEF improved significantly better in the emergency group than in the elective group, and the difference was statistically significant (*P* < 0.05). The myocardial infarct quality, VSM score, and ventricular wall motion abnormality score were significantly lower in the emergency group than in the elective group from 7 to 10 d after PCI; myocardial infarct quality, VSM score, and ventricular wall motion abnormality score improved in both groups at 3 months after PCI; and the degree of improvement of myocardial infarct quality and VSM score was significantly better in the emergency group than in the elective group (*P* < 0.05). *Conclusion*. Acute myocardial infarction patients with significant effect of emergency PCI treatment can be on their postmyocardial infarction left ventricular function, and in the treatment of coronary heart disease, myocardial infarction diagnosis has a certain reference value.

## 1. Introduction

Myocardial infarction is a result of myocardial injury and structural and functional changes in the myocardium caused by various factors, which leads to low ventricular pumping or filling function [1, 2]. In the last decade, as CMRI has become more popular in treatment practice, it has been found that patients who successfully undergo PCI have a “no-reflow” phenomenon that can be visualized on cardiac magnetic resonance [3]. Evidence from one study showed that the area of microcirculatory obstruction was highly overlapping with the area of intramyocardial hemorrhage IMHD and also indicated that myocardial tissue was more severely damaged by vascular damage and red blood cell spillage than microcirculatory obstruction [2]. CMRI is an important and accurate method for quantitative evaluation of infarct size, degree of wall permeability, and microvascular obstruction in acute myocardial infarction and left heart function and is an effective and safe test for patients with nonmagnetic stents [4]. The CMRI technique allows dynamic visualization of cardiac motion and ventricular wall contraction, scanning continuous short-axis left ventricular movies, measuring ventricular diastolic and ventricular systolic volumes, and providing morphological and functional parameters [5]. The intensity of myocardial tissue signal enhancement depends on blood flow, tissue perfusion, the size of the extracellular space, and the state of contrast distribution within the myocardium [6]. Myocardial infarction is mainly characterized by structural destruction of myocardial cells and microvascular damage, and myocardial tissue perfusion and myocardial cell membrane integrity can be detected by contrast Gd-DTPA first-pass perfusion method and delayed phase scan [7]. In myocardial injury, the cell membrane is damaged, Gd-DTPA enters the myocardial cells with delayed efflux, so it shows delayed enhancement, and the high signal area of delayed enhancement represents irreversible necrotic myocardium [8]. Based on this, we have conducted some exploration for the effect of CMRI assessment on the protective effect of coronary microcirculatory function after reperfusion of myocardial infarction, and the results of the research are now reported as follows.

## 2. Material and Methods

### 2.1. Research Object

According to the formula of cross-sectional survey sample size: *n* = *t*_*a*_^2^PQ/*d*^2^, *n* is the sample size, *P* is the prevalence of myocardial infarction, *Q* = 1 − *P*, *d* is the allowable error. *a* = 0.05, *t*_*a*_ = 1.96. The minimum sample size is 200 cases, and the actual sample size of 280 cases of myocardial infarction was included in this study. 13 cases were dropped due to transfer and moving. Cases and the rest were divided into the emergency group and the elective group of 140 cases each. Baseline information such as gender, age, and other information of patients in both groups had no effect on this study. The selected patients were all patients with myocardial infarction, and there were no shedders or dropouts at 3 months of follow-up.

### 2.2. Exclusion Criteria

Inclusion criteria: (1) meeting the diagnostic criteria for acute ST-segment elevation myocardial infarction in the Guidelines for the Diagnosis and Treatment of Acute ST-segment Elevation Myocardial Infarction [9] (ischemic chest pain episodes lasting more than 30 minutes that are not relieved by nitroglycerin; ECG with ST-segment elevation in two or more adjacent leads, limb leads ≥ 1 mm and chest leads ≥ 2 mm; or newly developed left bundle branch conduction block; serologic markers of myocardial necrosis were elevated at least twice the normal value), (2) acute myocardial infarction confirmed by coronary angiography, (3) direct PCI within 24 hours of onset, and (4) complete angiographic data. Exclusion criteria: (1) those who were uncooperative in the examination, poor compliance, unable to guarantee completion of the test, those with impaired consciousness and obvious intellectual impairment and mental abnormalities; (2) those with metal foreign bodies, such as metal prostheses, intraocular metal foreign bodies, intracranial aneurysm clamps, etc., those suffering from closed phobia, those with a history of myocardial infarction, history of PCI treatment, and history of coronary artery bypass grafting; (3) those affecting ST-segment changes in the ECG Factors: complete left bundle branch block, preexcitation syndrome, pacemaker ECG, etc., known severe peripheral vascular disease.

### 2.3. Methods

#### 2.3.1. PCI Treatment

Patients in the emergency group were treated with PCI immediately after admission (within 12 h after infarction). The elective group underwent PCI 6-8 d after infarction. The selection of the indication and timing of the procedure was determined by the treating physician according to the Chinese Guidelines for Percutaneous Coronary Intervention (2016) [10] and combined with the patient's condition.

#### 2.3.2. CMRI

Patients in both groups underwent MRI at 7-10 d and 3 months after myocardial infarction with a Philips Intera 1.5TMas-tr superconducting magnetic resonance imaging machine, with the patient in the supine position, using a chest lead cardiac gating technique and a respiratory monitoring device, and a fast breath-hold sequence scan to complete long-axis (four-chamber) and short-axis (two-chamber) cardiac cine MRI acquisition. The morphological structure of the heart was observed at the short-axis level using a fast spin-echo sequence.

### 2.4. Observation Indicators

All cases were analysed independently by 2 radiology professors using a 3D analysis package based on a 16-segment model. Ventricular wall motion abnormalities were scored semiquantitatively on a scale of 0 to 4 using cardiac MRI techniques (score 0: normal; score 1: hypokinesis; score 2: no motion; score 3: paradoxical motion; score 4: ventricular wall tumour formation). The end-diastolic and end-systolic left ventricular wall contours were traced manually, and end-diastolic volume (EDV), end-systolic volume (ESV), and ejection fraction (EF) were calculated. Perfusion defects were analysed by computer-assisted volumetric method (CAVM) and visual scoring method (VSM) on first-pass as well as delayed perfusion imaging, respectively. Infarcted myocardial volumes were evaluated by CAVM with layer-by-layer manual tracing of delayed intensification contours and computer-assisted calculation.

### 2.5. Statistical Analysis

All statistical data in this study were entered into excel software by the first author and the corresponding author, respectively, and the statistical processing software was SPSS25.0 for calculation. Repeated measures analysis of variance between groups was used to measure the measurement expressed as mean ± standard deviation (*X* ± *S*). material. Count data expressed as a percentage (%) were tested by *χ*^2^. Univariate and logistic multivariate regression analyses were used to compare the influencing factors, and the risk factors with significant differences were screened. Univariate and logistic multivariate regression analyses were used to compare the influencing factors, and the risk factors with obvious differences were screened. The statistical significance was *P* < 0.05.

## 3. Results

### 3.1. Comparison of General Information

The comparison of general data such as gender, mean age, body mass index, and NYHA classification between the two groups was not statistically significantly different by *t*-test and chi-square test (*P* > 0.05), see Table 1.

### 3.2. Infarcted Myocardial Mass, VSM Score, and Ventricular Wall Motion Abnormality Score

Myocardial infarct quality, VSM score, and ventricular wall motion abnormality score were significantly lower in the emergency group than in the elective group from 7 to 10 d after PCI; myocardial infarct quality, VSM score, and ventricular wall motion abnormality score improved in both groups at 3 months after PCI; and myocardial infarct quality and VSM score improved significantly better in the emergency group than in the elective group (*P* < 0.05), see Figure 1.

### 3.3. Myocardial Microcirculatory Injury

The difference between peak troponin T and peak BNP in each group by rank sum test was not statistically significant by comparison, whereas in the comparison of LVEF% mean values, it was found that the larger LVEF% mean values in the emergency group were statistically significant compared with the elective group (*P* < 0.05), see Figure 2.

### 3.4. Comparison of Cardiac Function Indexes

There was no statistically significant difference in the comparison of cardiac function indexes between the two groups of patients from 7 to 10 d after surgery (*P* > 0.05). The differences in hemodynamics (CO, CI, SV, SI, LVSW1, and LCW) measured at different times between the two groups after 3 months of surgery were significant; patients in the emergency group had significantly lower EDV and ESV than those in the elective group at 7 ~ 10 d postoperatively; EDV, ESV, and LVEF improved in both groups after 3 months, while EDV, ESV, and LVEF improved significantly better in the emergency group than in the elective group; and the difference was statistically significant (*P* < 0.05), see Figure 3.

### 3.5. Hemodynamic Comparison

There was no statistically significant difference in the hemodynamic comparison between the two groups (*P* > 0.05). LVESV, GEDVI, and LVEF were significantly improved and significantly better in the emergency group than in the elective group in both groups, with statistically significant differences in comparison (*P* < 0.05), see Figure 4.

## 4. Discussion

After acute myocardial infarction, restoration of myocardial perfusion by opening the criminal vessel as soon as possible through interventional or thrombolytic therapy is the main treatment currently aimed at reducing the infarct size as well as mortality [11]. However, with the opening of the epicardial vessels, 50% of patients still suffer from ischemia at the level of myocardial microcirculation, i.e., the “no-reflow phenomenon” [12]. The pathological mechanism is the blockage of the microvascular lumen by platelets, leukocyte debris and microthrombi, edema of the endothelium, or compression by edema of the myocardial tissue, as well as the pathological inflammatory response, vasospasm due to thrombus, and vasoconstrictor secreted by the endothelium [13]. Persistent myocardial ischemia and massive necrosis due to no recurrent flow are important determinants of death and other adverse events after infarction [14]. However, in recent years, it has been found that prolonged microcirculatory impairment with severe tissue ischemia and hypoxia can lead to destruction of capillary walls and spillage of red blood cells from the vessels into the tissue interstitium, a more severe form of reperfusion injury [15].

In terms of left ventricular function, EDV, ESV, and LVEF improved at 3 months after PCI, but the degree of improvement was significantly better in the emergency group than in the elective group. It suggests that all eligible patients should be opened to coronary vessels as early as possible to achieve myocardial reperfusion. Emergency PCI can rapidly open infarct-related vessels, TMI blood flow can mostly reach grade 3, and myocardial tissues can be effectively perfused, which can reduce the scope of infarction, save dying myocardial cells, reduce edema of peri-infarct tissues, and control the development of ventricular remodeling, thus protecting and improving cardiac function [16, 17]. However, a significant proportion of patients with myocardial infarction still miss the optimal time to open the vessel for various reasons and opt for elective PCI [18]. Elective PCI delays reperfusion time, and some myocardium undergoes irreversible necrosis, which is not conducive to stopping the progression of ventricular remodeling [19–22].

There are some limitations of this study: the samples selected were from our hospital inclusion exclusion are subjective and the number is small, and the findings may not be generalizable; we failed to study in depth the treatment effect of patients with myocardial infarction in long follow-up.

In conclusion, the effect of emergency PCI in patients with acute myocardial infarction is significant and can be used for their postmyocardial infarction left ventricular function, which has a certain reference value in the treatment of coronary heart disease myocardial infarction diagnosis.

## Figures and Tables

**Figure 1:** Comparison of infarct quality, VSM score, and ventricular wall motion abnormality score detected by CMRI (The data of myocardial infarct quality, VSM score, and ventricular wall motion abnormality score were entered into the computer database by the first author and checked and corrected by the corresponding author to ensure the completeness and accuracy of the data. The measures were expressed as mean ± standard deviation using *t*-test and found that myocardial infarct quality (a), VSM score (b), and ventricular wall motion abnormality score (c) improved in both groups 3 months after PCI, and the improvement of myocardial infarct quality and VSM score in the emergency group was significantly better than that in the elective group (*P* < 0.05)).

**Figure 2:** Comparison of myocardial microcirculatory injury (Myocardial microcirculatory injury data were entered into the computer database by the first author and checked and corrected by the corresponding author to ensure the completeness and accuracy of the information. The measurement data were expressed as mean ± standard deviation using *t*-test and found that the difference between peak troponin T and peak BNP in each group by rank sum test was not statistically significant by comparison, while in the comparison of LVEF% mean value was found to be statistically significant (*P* < 0.05) in the emergency group with larger LVEF% mean value compared with the elective group).

**Figure 3:** Comparative comparison of cardiac function indexes (Data of cardiac function indexes were entered into the computer database by the first author and checked and corrected by the corresponding author to ensure the completeness and accuracy of the information. The measurement data were expressed as mean ± standard deviation using *t*-test and found that the hemodynamics (CO, CI, SV, SI, LVSW1, and LCW) measured at different times in the two groups were significantly different after 3 months of surgery; patients in the emergency group had significantly lower EDV and ESV than the elective group at 7-10 d after surgery; and EDV, ESV, and LVEF improved in both groups after 3 months, while the emergency group EDV, ESV, and LVEF improved significantly better than the elective group, and the difference was statistically significant (*P* < 0.05)).

**Figure 4:** Hemodynamic comparison between the two groups (Hemodynamic index data were entered into the computer database by the first author and checked and corrected by the corresponding author to ensure the completeness and accuracy of the information. The measures were expressed as mean ± standard deviation using *t*-test and found that LVESV (a), GEDVI (b), and LVEF (c) were significantly improved and significantly better in the emergency group than in the elective group in both groups, with statistically significant differences in comparison (*P* < 0.05)).

**Table 1:** Comparison of general information between the two groups (*n*, ($\bar{x}\pm s$)).

Group	Gender (male/female)	Average age (years)	Body mass index (kg/m^2^)	NYHA classification		
				I	II	III ~ IV
Elective group (140)	73/67	56.63 ± 8.32	26.31 ± 3.67	50	43	47
Emergency group (140)	72/68	56.62 ± 8.31	26.33 ± 3.25	52	42	46
*χ* ^2^/*t*	0.014	0.010	-0.048	0.062	0.017	0.016
*P*	0.905	0.992	0.962	0.804	0.897	0.900

## Data Availability

The experimental data used to support the findings of this study are available from the corresponding author upon request.
